The article "The Ratio of Circulating Regulatory T Cells (Tregs)/Th17 Cells Is Associated with Acute Allograft Rejection in Liver Transplantation" was retracted in 2019. Reasons: lack of ethics approval or compliance; missing or withdrawn patient consent; ethical violations by an author; concerns about the data.

# The Ratio of Circulating Regulatory T Cells (Tregs)/Th17 Cells Is Associated with Acute Allograft Rejection in Liver Transplantation

**DOI:** 10.1371/journal.pone.0112135

**Published:** 2014-11-05

**Authors:** Ying Wang, Min Zhang, Zhen-Wen Liu, Wei-Guo Ren, Yan-Chao Shi, Yan-Ling Sun, Hong-Bo Wang, Lei Jin, Fu-Sheng Wang, Ming Shi

**Affiliations:** 1 Research Center for Liver Transplantation, Beijing 302 Hospital, Peking University Health Science Center, Beijing, China; 2 Research Centre for Liver Transplantation, Beijing 302 Hospital, Beijing, China; 3 The Third Xiangya Hospital of Central South University, Changsha, China; 4 Research Center for Biological Therapy, Beijing 302 Hospital, Beijing, China; UNIFESP Federal University of São Paulo, Brazil

## Abstract

CD4^+^CD25^+^FoxP3^+^ regulatory T cells (Tregs) and Th17 cells are known to be involved in the alloreactive responses in organ transplantation, but little is known about the relationship between Tregs and Th17 cells in the context of liver alloresponse. Here, we investigated whether the circulating Tregs/Th17 ratio is associated with acute allograft rejection in liver transplantation. In present study, thirty-eight patients who received liver transplant were enrolled. The patients were divided into two groups: acute allograft rejection group (Gr-AR) (n = 16) and stable allograft liver function group (Gr-SF) (n = 22). The frequencies of circulating Tregs and circulating Th17 cells, as well as Tregs/Th17 ratio were determined using flow cytometry. The association between Tregs/Th17 ratio and acute allograft rejection was then analyzed. Our results showed that the frequency of circulating Tregs was significantly decreased, whereas the frequency of circulating Th17 cells was significantly increased in liver allograft recipients who developed acute rejection. Tregs/Th17 ratio had a negative correlation with liver damage indices and the score of rejection activity index (RAI) after liver transplantation. In addition, the percentages of CTLA-4^+^, HLA-DR^+^, Ki67^+^, and IL-10^+^ Tregs were higher in Gr-SF group than in Gr-AR group. Our results suggested that the ratio of circulating Tregs/Th17 cells is associated with acute allograft rejection, thus the ratio may serve as an alternative marker for the diagnosis of acute rejection.

## Introduction

Despite the use of potent immunosuppressive agents, acute rejection (AR) remains a major cause of early allograft loss and an obstacle for long-term allograft survival. The hallmarks of acute rejection include infiltration of T lymphocytes, monocytes, and other inflammatory cells [1], [2]. Laboratory and clinical investigations have indicated that CD4^+^CD25^+^FoxP3^+^ regulatory T cells (Tregs) are one of the major cell types responsible for the immune responses to alloantigens. Tregs activation is involved in the prevention of rejection, the induction and maintenance of peripheral tolerance of the allograft [3], and the support of allograft survival [4]–[6]. Several other studies indicated that Tregs are an essential element of the immunoregulatory pathway which induces peripheral allograft tolerance [7], [8], that the frequency of circulating Tregs is significantly decreased during acute rejection [9], and that the transfer of Tregs pre-stimulated *in* *vitro* can protect skin and cardiac allografts from acute and chronic rejection [10], [11]. In clinical transplantation, T cells with the phenotypic characteristics of regulatory cells are detected in both the peripheral blood and within the graft itself [3], [12], [13]. In renal transplant recipients, grafts infiltrated with more Tregs display much longer survival [7], [14]. Pediatric patients who acquired operational tolerance after liver transplantation showed increased levels of circulating Tregs compared with patients who received immunosuppression [12]. Allograft tolerance in liver transplant recipients may be partly attributable to a higher frequency of circulating Tregs [9]. Therefore, an increased level of circulating Tregs may be beneficial for allograft survival.

Th17 cells are a subset of T helper cells which is characterized by the production of IL-17. Th17 cells have been suggested to play a role in allograft rejection in the context of organ transplantation [15]–[18]. A study reported that cardiac allografts infiltrated with Th17 cells underwent accelerated vascular rejection in Tbet−/− mice model [19]. IL-17, a potent proinflammatory cytokine, has been demonstrated to participate in allograft rejection [20]–[23]. It promotes cardiac allograft rejection by inducing the maturation, antigen presentation, and co-stimulatory capabilities of dendritic cells in mice [20]. In a corneal transplant model, mice with deficient IL-17 experienced delayed graft rejection compared to wild-type mice [24]. Blocking IL-17 promoted the maturation of dendritic cells, inhibited the proliferation of alloreactive T cells *in* *vitro*, and prolonged the survival time of vascularized cardiac allografts *in* *vivo* [19], [20]. IL-17 neutralization inhibits acute, but not chronic, vascular rejection in mice [17], [25]. Clinical evidence showed that the level of IL-17 in the blood is positively correlated with acute allograft rejection in the renal [21], [26] and the liver [22] transplant recipients. Graft infiltrated with Th17 cells is associated with a faster destruction of allograft in renal transplant patients [27], [28].

The aforementioned evidence suggests that Tregs cells have a protective effect against graft rejection, whereas Th17 cells play an essential role in promoting graft rejection. The differentiation pathways of Tregs and Th17 cells are known to be antagonistic [29], [30], and Tregs can be converted into Th17 cells under inflammatory conditions [31]. However, the relationship between Tregs and Th17 cells is yet to be fully understood in the context of transplant alloresponse. Further validation is necessary to determine whether the balance between circulating Tregs and Th17 cells may be used as a predictor for the outcome of transplantation. This study is aimed to investigate the dynamics of Tregs/Th17 ratio in liver transplant recipients with or without post-operative rejection, and to assess whether Tregs/Th17 ratio may serve as an alternative marker for the diagnosis of acute rejection.

## Materials and Methods

### Patients

The study protocol was approved by the institutional review board of Beijing 302 hospital. All participants provided written informed consent to participate in this study. Thirty-eight patients were enrolled in our hospital for this study. All participants received a first cadaveric liver transplantation with an identical or compatible blood-group graft. Based on clinical and biochemical indicators as well as pathologic diagnosis, the patients were divided into two groups: acute allograft rejection group (Gr-AR, n = 16) and stable allograft liver function group (Gr-SF, n = 22). The histopathologic diagnosis of acute allograft rejection was defined according to Banff criteria [32]. Acute rejection and stable allograft liver function were defined as previously described [33]. All patients received conventional immunosuppressive agents after liver transplantation, such as tacrolimus, steroids (prednisolone) and mycophenolate mofetil (MMF). The dose of tacrolimus was adjusted when acute rejection was diagnosed. Patients with HBV infection received prophylactic therapies with hepatitis B immune globulin (HBIG) plus nucleos(t)ide analogues (NAs). The blood samples were obtained from all patients prior to transplant and at the following timepoints after transplantation: 1, 2, 3, 4, 8, 12 weeks. In addition, the blood samples and allograft biopsy tissues were obtained at the time of presenting worsening liver function test results and/or symptoms suggestive of acute rejection after liver transplantation. The clinical characteristics of these subjects were listed in Table 1.

**Table 1:** Characteristics of participants.

Parameters	Gr-AR	Gr-SF
	n = 16	n = 22
Age (Mean±SD)	51±9	49±11
Gender (M/F)	11/5	15/7
Primary etiology		
HBV	10	15
HCV	2	3
HBV+HCV	1	2
Alcohol	3	2

### Flow cytometric analysis

The phycoerythrin (PE)-conjugated anti-IL-17A and fluorescein isothiocyanate (FITC)-conjugated anti-FoxP3 were purchased from eBioscience (San Diego, CA), and all other antibodies used in flow cytometry were from BD Biosciences (San Jose, CA). For immunostaining of intracellular IL-17A, two samples of freshly heparinized peripheral blood (200 µL each) were incubated for 6 hours with phorbol-12-myristate-13-acetate (PMA, 300 ng/mL, Sigma-Aldrich, St. Louis, MO) and ionomycin (1 µL/mL, Sigma-Aldrich) in 800 µL of RPMI 1640 medium supplemented with 10% fetal calf serum. Monensin (0.4 µM, BD PharMingen) was added during the first hour of incubation. Then cytofix/cytoperm kit (BD PharMingen), anti-CD3, anti-CD8, anti-IL17, and anti-IFN-γ antibody (mAb) were used in one sample, whereas anti-CD4, anti-CD25, and anti- FoxP3 mAb were used in the other sample according to the manufacturers’ protocols. For Tregs analysis, anti-CD4, anti-CD25, and anti-HLA-DR mAb were added to 200 µL freshly heparinized blood sample, and then the sample was permeabilized and fixed using fix/perm kit (eBioscience) according to the manufacturer’s instructions. After permeabilization, cells were incubated with anti-FoxP3, anti-CTLA-4, and anti-Ki67 mAb. The stained cells were acquired on a FACSCalibur (BD Biosciences) and analyzed using FlowJo software (Tritar, USA).

### Immunohistochemistry

Biopsy specimens from 16 patients with acute rejection were collected and used in immunochemical staining with antiFoxP3 (eBioscience) and anti-IL-17 (R&D Systems). Formalin-fixed, paraffin-embedded liver tissues were cut into 5 µm sections and placed on polylysine-coated slides. Antigen retrieval was achieved via pressure cooking for 10 min in citrate buffer (pH 6.0). Endogenous peroxidase activity was blocked with 0.3% H_2_O_2_. The sections were then incubated with anti-FoxP3 or anti-IL-17 antibodies for overnight at 4°C. 3-amino-9-ethyl-carbazole (red color) was used as a substrate, and hematoxylin was used in the subsequent counterstaining.

### Statistical analysis

SPSS 16.0 software (SPSS, Chicago, IL, USA) was used for all statistical analyses. The data were presented as means ± SD. Mann-Whitney nonparametric *U*-test was applied to comparisons between 2 groups. Spearman’s rank test was used to analyze the association between the severity of allograft tissue injury and Tregs frequency, Th17 cell frequency, or Tregs/Th17 ratio. Chi-square-test was used to assess the difference among clinical data. A value of *P*<0.05 was considered to be statistically significant.

## Results

### The patterns of Tregs and Th17 cell frequencies and Tregs/Th17 ratio in transplant recipients with acute rejection

We investigated Tregs and Th17 cell frequencies and Tregs/Th17 ratio in all participants after liver transplantation. We collected the values of Tregs, Th17 cells and Tregs/Th17 ratio in Gr-SF and Gr-AR in the period prior to a rejection or at the onset of acute rejection after liver transplantation, and compared the values in Gr-SF group to those in Gr-AR group. Flow cytometry was used to analyze Tregs and Th17 frequencies in peripheral blood in all patients after liver transplantation. The results showed that during the period preceding rejection, the frequencies of Tregs, Th17 cells, and the Tregs/Th17 ratio have not significant differences between two groups. At the period onset of acute rejection, however, the frequency of Tregs was significantly higher in Gr-SF than in Gr-AR (*P*<0.01), but the frequency of Th17 was significantly lower in Gr-SF than in Gr-AR (*P*<0.01), yielding a significantly higher Tregs/Th17 ratio in Gr-SF than in Gr-AR (*P*<0.01). In addition, the frequency of IL-17/IFN-γ producing CD4^+^ T cells (IL-17^+^IFN-γ^+^) was higher in Gr-AR than that in Gr-SF (*P*<0.05) (Fig. 1A, B).

**Figure 1:** The distribution of Tregs and Th17 cells in the peripheral blood and in the grafts of patients with acute allograft rejection. (A) Representative profiles of Tregs and Th17 cells in peripheral blood collected using fluorescence-activated cell sorter (FACS). (B) The frequency of Tregs and Tregs/Th17 ratio were significantly higher in Gr-SF than in Gr-AR. On the contrary, the frequency of Th17 cells was significantly lower in Gr-SF than in Gr-AR. In addition, the frequency of IL-17^+^IFN-γ^+^ cells was lower in Gr-SF than in Gr-AR. (C) To evaluate the distribution pattern of Tregs and Th17 cells in allografts with acute rejection, we examined the infiltration of Tregs and Th17 cells using immunohistochemical staining. Anti-FoxP3^+^ and anti-IL-17 antibodies were used on paraffin embedded biopsy samples which were obtained from allograft with acute rejection. The results showed extensive infiltration of Tregs (red) and Th17 cells (red). Original magnification, ×400. (D) One representative patient with acute allograft rejection was followed-up for 12 months after liver transplantation. The dynamics of Tregs and Th17 cell frequencies were depicted during the follow-up period (the black line represents Th17 cells frequency; the blue line the Tregs frequency; and the red line Tregs/Th17 ratio). ARS: Acute rejection subsided.

To investigate the distribution patterns of Tregs and Th17 cells in acute rejection allografts, we next examined the infiltration of Tregs and Th17 cells in biopsy samples obtained from allografts in patients with acute rejection. Immunohistochemical staining was performed using anti-FoxP3^+^ and anti-IL-17 antibodies on paraffin embedded sections. Our results demonstrated an extensive infiltration of Tregs and Th17 cells in the acute reject allograft liver tissue (Fig. 1C). These findings, along with previously published data [34], suggested that Tregs may be involved in the regulation of alloreactive response in liver allograft tissue, but might be deficient in some patients. One representative patient with acute allograft rejection was followed up for 12 months after liver transplantation. The dynamics of Tregs and Th17 cell frequencies during the follow-up period was depicted in Figure 1D. The Th17 cell frequency exhibited a trend opposite to that of Tregs or Tregs/Th17 ratio. At the onset of acute rejection, Tregs frequency and Tregs/Th17 ratio were sharply decreased, whereas Th17 cell frequency was dramatically increased. Interestingly, as the rejection subsided, the frequencies of Tregs and Th17 cells were both restored to levels close to those before rejection.

### The correlation between Tregs/Th17 ratio and the biochemical indices of liver damage

Little is known about the association between the balance of Tregs/Th17 and the liver damage in liver transplant recipients. Therefore, we analyzed the correlation of Tregs/Th17 ratio and the biochemical indices of liver damage, such as alanine amino transferase (ALT), aspartate amino transferase (AST), alkaline phosphatase (ALP) and gamma-glutamyl transpeptidase (GGT), in the 16 patients during the acute allograft rejection episode. Negative correlations were observed between Tregs/Th17 ratio and the levels of ALT (r = −0.668, *P* = 0.005), AST (r = −0.541, *P* = 0.031), ALP (r = −0.518, *P* = 0.039), and GGT (r = −0.764, *P* = 0.001) (**Fig. 2**). These results indicated that Tregs/Th17 ratio may be used as an alternative indicator for the diagnosis of liver damage in liver transplant recipients.

**Figure 2:** Tregs/Th17 ratio is correlated with the serum levels of ALT, AST, ALP and GGT. We analyzed the correlation between the ratio of circulating Tregs/Th17 and the biochemical indices for liver damage, ALT, AST, ALP and GGT, in the 16 patients with acute allograft rejection. Negative correlations were found between the ratio of circulating Tregs/Th17 and the levels of ALT, AST, ALP, and GGT (*P*<0.05).

### Tregs frequency, Th17 cell frequency, and Tregs/Th17 ratio is correlated with rejection activity index (RAI)

To confirm whether Tregs and Th17 cells were associated with liver allograft rejection, we analyzed the correlation between the rejection activity index (RAI) and the frequencies of circulating Tregs and Th17 cells. We found that Tregs/Th17 ratio (r = −0.859, *P*<0.001) and the level of Tregs (r = −0.867, *P*<0.001) had a negative correlation with RAI, whereas the level of Th17 cells showed a positive correlation with RAI (r = 0.890, *P*<0.001) (**Fig. 3**). These results suggested that Tregs/Th17 ratio may serve as a biomarker for the diagnosis of acute rejection.

**Figure 3:** The frequency of Tregs, the frequency of Th17 cells, and Tregs/Th17 ratio are correlated with RAI. To confirm whether Tregs, Th17 cells and Tregs/Th17 were associated with the liver allograft rejection, we analyzed the correlation between RAI and the frequency of circulating Tregs, the frequency of circulating Th17 cells, and Tregs/Th17 ratio. We found that the Tregs level and Tregs/Th17 ratio had a negative correlation with RAI, whereas the Th17 cell level showed a positive correlation with RAI (*P*<0.01).

### The phenotypes of CTLA-4^+^, HLA-DR^+^, Ki67^+^ Tregs in liver transplant patients

To better understand the mechanism by which Tregs function in liver transplant recipients, some important molecules that regulate Tregs were analyzed. CTLA-4 is expressed by human Tregs and is also upregulated in T cells upon activation. We characterized the patterns of CTLA-4 expression in Tregs in all patients. The percentage of CTLA-4**^+^** Tregs was calculated as the percentage in total Tregs. The results showed that the frequency of CTLA-4^+^ Tregs was higher in Gr-SF group (35.5±18.9%) than in Gr-AR group (23.7±12.8%) (*P*<0.05). We also evaluated the activated (HLA-DR^+^) and proliferating (Ki67^+^) Tregs in peripheral blood in all patients. We found that the percentages of HLA-DR^+^ Tregs and Ki67^+^ Tregs were higher in Gr-SF (26.8±17.2%, 30.6±15.8%, respectively) than in Gr-AR (17.2±11.6%, 20.3±10.9%, respectively) (*P*<0.05) (**Fig. 4**). Such data suggested that more Tregs were in active and proliferating state in Gr-SF than in Gr-AR, and may facilitate the suppression of alloreactive responses in liver transplant recipients.

**Figure 4:** The phenotypes of CTLA-4^+^, HLA-DR^+^, Ki67^+^ Tregs in liver transplant patients. The activated and proliferative molecules on Tregs were detected in liver transplant patients. The results showed that the frequencies of CTLA-4^+^, HLA-DR^+^, and Ki67^+^ Tregs were higher in Gr-SF than in Gr-AR (all *P*<0.05). The above data suggested more Tregs were active and proliferating in Gr-SF than in Gr-AR in liver transplant recipients.

## Discussion

Many studies have demonstrated that CD4^+^CD25^+^FoxP3^+^ Tregs and Th17 cells are involved in the tolerance or rejection response in organ transplantation [17], [34]–[37]. The current study is designed to investigate the relationship between Tregs and Th17 cells in the context of alloresponse in liver transplant patients. The major finding of our study is that Tregs/Th17 ratio is associated with alloresponse after liver transplantation. Our data confirm that the frequency of circulating Tregs is significantly decreased, whereas the frequency of Th17 cells is significantly increased in liver allograft recipients with acute rejection, and that Tregs/Th17 ratio has a negative correlation with liver damage. To our knowledge, this is the first study to demonstrate an association between Tregs/Th17 imbalance and allografts rejection. These findings suggest that the ratio of circulating Tregs/Th17 may serve as an alternative marker for the diagnosis of acute rejection and for the evaluation of the immune status in liver transplant recipients.

Tregs are a unique subset of CD4^+^ T helper cells in that they control the responses of effector T-cells to prevent autoimmune reactions. Several studies show that Tregs can prevent rejection and promote the long-term survival of skin grafts in a mouse model [6], [38]. In clinical, Tregs have been reported to be associated with allograft tolerance in liver transplant recipients [9], [12]. The Th17 subset is involved in mediating autoimmune responses and regulating allograft rejection both in rat renal transplant models and human renal transplantation [39], [40]. In lung and heart transplantation, IL-17 has also been reported to be involved in allograft acute rejection [41], [42]. A recent study reported that the levels of circulating CD4^+^IL^−^17^+^ T cells are substantially higher in rejection group than in non-rejection group in liver transplant recipients, and the frequency of CD4^+^IL^−^17^+^ cells in peripheral blood is positively correlated with the rejection activity index [43]. Recent researches reported that a new subpopulation of CD161^+^ Treg is able to produce IL-17 and has both inflammatory and suppressive potentials [44], [45]. The functional and phenotypic characteristics of this subset in alloreactive response are worth further study.

The frequency of Tregs in Gr-AR is significantly lower; on the contrary, the frequency of Th17 cells in Gr-AR is significantly higher than that in Gr-SF. In addition, the frequency of circulating Tregs has a negative correlation with RAI, whereas the frequency of circulating Th17 cells has a positive correlation with RAI. These data indicate that the decreased levels of Tregs and increased levels of Th17 cells may be involved in the acute rejection episodes in liver transplantation. Histopathological results demonstrate that the allograft tissue with acute rejection is extensively infiltrated with Tregs and Th17 cells. These findings are consistent with that from Stenard’s study, which revealed increased intragraft Tregs during acute rejection [34]. Such data suggest that Tregs are mobilized to the site of immune activation and may participate in the regulation of alloreactive responses. However, the observation that acute allograft rejection can occur, even in the presence of Tregs, indicates that at least under some circumstances the mobilization of Tregs to the site is insufficient to effectively down-modulate the alloreactivity.

Next, we suggest the mechanism by which Tregs are involved in the rejection episodes. CTLA-4 is an inhibitory receptor expressed by both activated T cells and Tregs, and may be crucial for their activity. HLA-DR is a marker for T cell activation. Ki67 is a marker of T cell proliferation. In our results, the percentages of CTLA-4 and HLA-DR^+^ Tregs are significantly higher in Gr-SF than in Gr-AR. In addition, the level of Ki67^+^ Tregs is significantly higher in Gr-SF than in Gr-AR. In general, the increase in the frequencies of CTLA-4^+^ Tregs, HLA-DR^+^ Tregs, and Ki67^+^ Tregs following the alloreactive immunosuppression may facilitate Tregs to exert their suppressive function, and may reflect the restoration of their functions because these changes occurred in parallel with stable liver functions. However, we have not assessed the suppressive function of Tregs in stable versus acutely rejecting subjects, so cannot draw any conclusions about the functional relevance of these cells in preventing/ameliorating rejection and impacting transplant outcomes.

In conclusion, maintaining an appropriate balance between Tregs and Th17 cells is indispensable for the maintenance of stable liver function in transplant recipients. Tilting Tregs-Th17 equilibrium toward Tregs dominance may promote transplant tolerance. However, we carried out a small-scale observation study that is underpowered to draw firm conclusions about cause and effect between Treg/Th17 ratio and acute rejection. These findings should be the subject of further inquiry through a carefully conducted, larger, prospective study to determine whether Tregs/Th17 ratio can be used as a diagnosis marker and whether it may serve as a potential therapeutic target to manage the acute rejection of liver allografts.
